# Study on the Effect of Self-Made Lifei Dingchuan Decoction Combined with Western Medicine on Cough Variant Asthma

**DOI:** 10.1155/2022/9803552

**Published:** 2022-09-12

**Authors:** Jiachun Li, Ziliang Huang, Keying Li, Xiaoyun Jian, Binghui Liang

**Affiliations:** ^1^Department of Respiratory Medicine, Foshan Hospital of Traditional Chinese Medicine, Guangzhou University of Traditional Chinese Medicine, Foshan, Guangdong 528000, China; ^2^The Third School of Clinical Medicine, Guangzhou University of Chinese Medicine, Guangzhou, Guangdong 510145, China; ^3^Department of Traditional Chinese Medicine, The Sixth Affiliated Hospital of Guangzhou Medical University, Qingyuan People's Hospital, Qingyuan, Guangdong 511518, China; ^4^The Eighth School of Clinical Medicine, Guangzhou University of Chinese Medicine, Foshan, Guangdong 528000, China

## Abstract

**Aims:**

To observe the clinical efficacy of self-made Lifei Dingchuan decoction combined with western medicine in the treatment of cough variant asthma (phlegm-heat accumulation in the lung syndrome).

**Materials and Methods:**

The clinical data of 90 patients with cough variant asthma who were hospitalized in the Department of Respiratory Medicine of our hospital from January 2020 to April 2022 were selected as the research objects, and they were equally divided into the observation group and the reference group according to different treatment methods, 45 cases in each group. The group was treated with traditional montelukast sodium chewable tablet and salmeterol fluticasone mixed powder inhalation, and the observation group was treated with self-made Lifei Dingchuan decoction on the basis of the control group, saturation, pH, partial pressure of oxygen in arterial blood, partial pressure of carbon dioxide, length of stay, and hospitalization costs.

**Results:**

After the patients underwent self-made Lifei Dingchuan decoction, there were significant differences between the observation group and the reference group in terms of heart rate, respiratory rate, blood oxygen saturation, pH value, arterial blood oxygen partial pressure, carbon dioxide partial pressure, and within the group. There was a statistical difference (*P* < 0.05). The adverse reactions in patients with cough variant asthma after treatment showed that the red throat, shortness of breath, chest tightness, and dry mouth in the observation group were significantly different from those in the control group (*P* < 0.05). After investigation, follow-up, and statistics, the hospitalization time, hospitalization cost, asthma exacerbation control time, effective rate, and recurrence rate were compared between the two groups, and the differences between the two groups were statistically significant (*P* < 0.05).

**Conclusion:**

The study on the clinical efficacy and low hospitalization cost of the self-prepared lung and asthma-restorative soup in patients with cough variant asthma significantly improved the patients' arterial oxygen saturation, acid-base value, arterial partial pressure of oxygen, and partial pressure of carbon dioxide and effectively controlled the heart rate and respiratory rate with high safety, which is worth further promotion.

## 1. Introduction

Cough variant asthma (CVA) is one of the most frequent respiratory diseases. Cough variant asthma is a specific type of asthma in which cough is the only or main clinical manifestation without obvious signs or symptoms such as wheezing and shortness of breath, but with airway hyperresponsiveness. The main manifestation is an irritating dry cough [1]. The cough is usually more intense, with nocturnal cough as its important feature, and severe cases are accompanied by chest tightness and shortness of breath [2]. The incidence of CVA has been increasing year by year in recent years, and 41.95% of all chronic cough patients in China in 2021 were further developed from CVA [3]. It is highly likely that nearly 30% of patients with CVA without clinical diagnosis and treatment will eventually develop and evolve into typical asthma [4].

At present, it is believed that the pathogenesis of this disease is similar to that of typical asthma. The etiology includes genetic factors, allergic factors, infectious factors, and a series of physical and chemical factors. It has the physiological and pathological characteristics of chronic airway inflammation, airway remodeling, and airway hyperresponsiveness. It may be related to the sensitization of cough receptors and the increased wheezing threshold. Commonly used therapeutic drugs include inhaled corticosteroids (ICS), leukotriene receptor antagonists, bronchodilators, antihistamines, mast cell membrane stabilizers, macrolides, expectorants, and immunomodulators and have curative effect on CVA, but long-term use will produce side effects, and the recurrence rate is high once it is stopped. In addition, nondrug treatment methods such as specific immunotherapy will be used clinically. Although it is expected to cure the disease, the course of treatment is long, and the compliance of children is poor.

Cough variant asthma belongs to the category of cough, whooping cough, and pharyngogenic cough in Chinese medicine. In recent years, TCM has conducted some research on its mechanism and treatment, and certain progress has been made [5]. Traditional Chinese medicine has accumulated rich experience in the diagnosis and treatment of pulmonary cough and asthma and has formed a large number of effective prescriptions and medicines [6]. Modern TCM studies have shown significant efficacy in improving the clinical symptoms of CVA patients [7]. The results of Chinese medicine compound for the treatment of cough variant asthma suggest that it has a certain inhibitory effect on the pathological changes such as airway hyperreactivity, chronic allergic inflammation of airways, and bronchospasm in cough variant asthma [8].

## 2. Material and Methods

### 2.1. Research Object

This study included 90 patients with cough variant asthma who were hospitalized in the Department of Respiratory Medicine of our hospital from January 2018 to April 2022 as the research subjects, and were divided into an observation group and a reference group with 45 cases in each group. The age group is between 18 and 65 years old. Western medicine diagnostic criteria for cough variant asthma: referring to the 2016 Guidelines for the Diagnosis and Prevention of Bronchial Asthma by the Respiratory Group of the Chinese Medical Association, the diagnostic criteria for CVA were formulated: (1) cough persisted for >4 weeks, often during exercise and at night and (or) early morning onset or aggravation, mainly dry cough without wheezing; (2) no signs of clinical infection or ineffective after prolonged antibiotic treatment; (3) effective antiasthma drug diagnostic treatment; (4) to exclude chronic cough caused by other causes; (5) positive bronchial provocation test and (or) PEF day − to − day variability rate (continuous monitoring for 2 weeks) ≥ 13%; (6) personal or first- and second-degree relatives with a history of allergic diseases or allergen test positive. As there is no unified standard for TCM syndrome differentiation of cough variant asthma in China, the TCM diagnostic criteria are based on preliminary clinical observation and review of literature on cough variant asthma syndrome research in recent years. The national planning textbooks “Traditional Chinese Medicine” and “Traditional Chinese Medicine Clinical Diagnosis and Treatment Guidelines-Cough Variant Asthma” published in “Journal of Traditional Chinese Medicine” in 2016 [9] formulate the TCM diagnostic criteria for cough variant asthma: (1) recurrent cough, it was paroxysmal and aggravated at night, in the morning or after activities; (2) expectoration with thick yellowish sputum. (3) Throat red (swollen), shortness of breath, chest tightness, dry mouth, dry stool (or) constipation, yellow urine, red tongue, and yellow greasy coating.

### 2.2. Include Exclusion Criteria

Inclusion criteria [9]: (i) meeting the above diagnostic criteria for cough variant asthma in Western medicine, meeting the diagnostic criteria in TCM and the TCM evidence of phlegm-heat in the lung; (ii) no obvious signs of infection at the time of inclusion in the trial, informed consent of the legal guardian to be tested; (iii) voluntary cooperation with the study, hospitalization days > 1 d. Exclusion criteria: (i) combined with other primary diseases of the lung, combined with serious primary diseases of the heart, liver, kidney, and hematopoietic system, psychiatric patients diseases, and psychiatric patients; (ii) those with other pathologies that reduce the likelihood of enrollment or complicate enrollment according to the investigator's judgment, those who had already taken Chinese and Western medicine for cough within 12 hours before the visit; (iii) those who were participating in clinical trials of other drugs and those with poor compliance that could easily cause shedding.

### 2.3. Methods

The reference group was treated with nasal catheter oxygen and conventional montelukast sodium tablets and salmeterol fluticasone mixed powder inhaler and oral montelukast sodium (Merck Sharp & Dohme Limited National Quota J20130054). Dosage: 10 mg/dose, 1 time daily, nightly at bedtime. Salmeterol fluticasone mixed powder inhaler, one inhalation in the morning and one in the evening every day, after the cough improved to once daily inhalation, the course of treatment for 1 month. In the observation group, the treatment was based on the control group, i.e., 10 g of roasted ephedra, 10 g of dilaemon, 10 g of bitter almonds, 10 g of scape seeds, 10 g of perilla seeds, 10 g of semen, 10 g of Qianhu, 10 g of mulberry bark, 10 g of Scutellaria, and 10 g of Yujin. During the treatment period, all other Chinese and Western medicine drugs for CVA were stopped. Patients were advised to prevent colds, eat a light diet, relax their emotions, exercise appropriately, avoid eating fatty, sweet, greasy and sizzling products, avoid raw and cold food, and avoid contact with any allergens as much as possible.

### 2.4. Statistical Analysis

SPSS 27.0 statistical software was used for analysis. Count data were expressed as the number of cases, and differences between the three groups were compared using chi-square test. If the measurement data obeyed normal distribution and the variance between the groups was the same, the data were expressed as mean ± standard deviation, and the differences between groups were compared using one-way ANOVA, and if the sample our data did not meet several conditions mentioned above, the data were expressed as median/interquartile spacing, and the comparison between the three groups was done using multiple independent sample our rank sum test (Kruskal-Wallis *H* test) with the test level *a* = 0.05.

## 3. Results

### 3.1. Baseline Data Comparison

The average age, gender, and common causes of patients in the observation group were not significantly different from those in the reference group, and the differences were not statistically significant (*P* > 0.05) (see Table 1).

### 3.2. Evaluation of Clinical Efficacy

There were statistically significant differences in heart rate, respiratory rate, oxygen saturation, acid-base value, arterial partial pressure of oxygen, and partial pressure of carbon dioxide between groups and within groups in the observation group and the reference group (*P* < 0.05). This result indicates a better clinical efficacy (see Figure 1).

### 3.3. Treatment Safety Evaluation

Drug toxicities after treatment in patients with cough variant asthma showed that symptoms such as red throat, shortness of breath, chest tightness, and dry mouth in the observation group were significantly different from those in the control group (*P* < 0.05). This result indicates a better treatment safety (see Figure 2).

### 3.4. Treatment Benefit Analysis

There were statistically significant differences between the two groups in terms of length of stay, hospital costs, time to control asthma exacerbation, efficiency, and recurrence rates (*P* < 0.05). This result indicates a better treatment benefit score for the treatment (see Figure 3).

## 4. Discussion

Most scholars believe that similar to typical asthma, on the one hand, the patient's own congenital constitution, “genetic quality,” immune status, mental state, health status, and other subjective factors, in addition to allergens, bacterial and viral infections, changes in climate, excessive exercise, occupational environment, and food and drugs, may be factors that promote the occurrence, and the pathogenesis of CVA is complex and clinically unclear, and studies have found that CVA and typical asthma have similar pathological features [10], such as the presence of specific inflammatory patterns and airway remodeling [12]. CVA patients only cough without wheezing, and there are nowadays three explanations for this phenomenon: the degree of ASR is lower in CVA compared to asthma, the wheezing threshold of CVA causing wheezing, and the coughing receptor sensitivity is also increased [13]. The bronchoconstriction reflex and the cough reflex are two interrelated and independent types of reflexes, and most of their cough receptors are present in the patient's airways, which are physically stimulated by the deformation of the airways due to bronchoconstriction and chemically stimulated by inflammatory mediators [14]. This causes the clinical symptoms of cough in patients, and the absence of cough receptors in the small airways will only result in contracture of the airways during an asthma attack, which will result in wheezing symptoms and croup in the lungs [15].

CVA is a specific type of asthma with chronic cough as the main clinical symptom, and its physiopathology is characterized by airway hyperresponsiveness, chronic airway inflammation, and airway remodeling. The pathogenetic factors are not clear, but are currently thought to be closely related to genetic factors, infectious factors, allergic factors, and some physicochemical factors. Because its clinical symptoms sometimes manifest only as cough, parents are very likely to ignore it or treat it as a simple cough, resulting in failure to treat or mistreatment and further development of typical asthma. Western medical treatment is similar to that of bronchial asthma and is graded. Commonly used drugs include low doses of ICS, leukotriene receptor antagonists, B2 agonists, and H2 receptor antagonists. Long-term use of hormones can produce many adverse effects, such as affecting the people's growth and development, bone metabolism, and immune function. Inhaled glucocorticoids can also cause oral Candida infections. Many scholars now believe that leukotriene receptor antagonists have comparable efficacy with ICS and advocate the use of leukotriene receptor antagonists instead of inhaled glucocorticoids as the drug of choice during cough variant asthma exacerbations. However, montelukast sodium as a representative drug of leukotriene receptor antagonists also has some problems, such as being more expensive and producing side effects such as allergy, diarrhea, and headache. In contrast, Chinese herbal medicine has the advantages of being cheaper and having fewer adverse effects when taken for a long time to treat this disease.

We studied that phlegm-heat-contained lung disease is a common type of this disease, once sick, the disease evil is easy to turn heat from Yang, so having the most heat evidence, whenever the regulation is not proper, it is easy to feel the external evil, and the external evil inside turns fire into heat [16]. The lung is a delicate organ with a clear deficiency, and it is not resistant to phlegm and heat, so the lung loses its ability to declaim and descend, resulting in cough due to Qi rebellion [17]. With deficiencies in the lungs, spleen, and kidneys, prolonged illness leads to deficiency, irregular elevation of the lungs, failure of the spleen to exercise and transport, and inability of the kidneys to transpire, resulting in stagnation of fluids, phlegm, and phlegm-heat interconnection and phlegm-qi rebellion, leading to cough [18]. Therefore, those with CVA with phlegm-heat-infused lung type often have recurrent cough, especially at night, and are often accompanied by real hot symptoms such as thick sputum, red face and lips, thirst, yellow urine, and constipation [19]. Based on our years of clinical experience, we combined the etiology and pathogenesis of CVA and established the treatment rules, focusing on clearing the lung and resolving phlegm, lowering qi, relieving cough, and calming asthma, and applied the self-prepared Rational Lung and Asthma Determining Tang to treat the evidence of phlegm and heat in the lung of CVA [20]. Self-designed Ruling Lung and Asthma Tang is derived from the combination of Self-designed Ruling Lung and Asthma Tang and Self-designed Ruling Lung and Asthma Tang [21]. This formula is the most typical one in the treatise on typhoid fever, and it is used to treat sun diseases in which sweating does not work or is misdirected as the lower evil qi enters the lung and turns into heat, which is smothered in the lung [22]. Pu Fu-Chou, a famous Chinese medicine practitioner, said that the self-prepared Rational Lung and Asthma Determining Soup can be used both to manage cold qi and to bring down fire qi, or for anyone with uncontrollable sweating [23]. It has therapeutic effects such as clearing heat and promoting lung-heating to stop coughing and calm asthma and is mainly used for coughing and shortness of breath caused by external internal heat and can be used for coughing and heat caused by wind and cold foreign to the interior [24]. It can be used for coughing and shortness of breath caused by heat entering the lungs from the wind and cold [25].

As a traditional ancient formula in Fushou Jingmen-Phlegm Gate, it is clearly stated in the original text that “specializes in treating snooze and asthma, with very rapid results [26].” It has the effect of promoting the lung and lowering qi, clearing heat, and resolving phlegm and can be used to treat asthma with phlegm-heat stagnation in the lung and can be used for asthmatic cough with croupy sound in the larynx or with vicious chills and fever, which is a symptom of wind-cold external bundle and phlegm-heat internal accumulation [27]. All of the self-prepared Ruling the Lung and Fixing Asthma Tang can treat the imbalance of the declination and purification of the lung qi and can also be clinically applied to some respiratory diseases with heat congestion in the lung [28]. The main pathogenic factor of Self-Designed Luling and Asthma Determining Tang is the external wind-cold evil, and Self-Designed Luling and Asthma Determining Tang is the phlegm evil, and this formula is formed by combining the two after cutting them according to experience, which can be effective in clearing the lung and resolving phlegm, lowering qi, and relieving cough and asthma.

Our study found that after the patients had undergone self-preparation of Ruling Lungs and Asthma Treatment Tang, there were significant differences in heart rate, respiratory rate, blood arterial oxygen saturation, acid-base value, arterial partial pressure of oxygen, and partial pressure of carbon dioxide between the observation group and the reference group, and there were statistically significant differences in adverse reactions after treatment in patients with cough variant asthma, including red throat, shortness of breath, chest tightness, and dry mouth in the observation group compared with the reference group. This indicates the clinical efficacy and low hospitalization cost of the self-prepared lung and asthma treatment for patients with cough variant asthma, which significantly improved the patients' arterial oxygen saturation, acid-base value, arterial partial pressure of oxygen, and partial pressure of carbon dioxide and effectively controlled the heart rate and respiratory rate with high safety. The main efficacy and mechanism of action of the self-prepared lung stabilization soup we studied are as follows: to treat the lung, we need to resolve the depression of lung qi and restore the normal elevation function of lung qi [29]. In this formula, sizzling ephedra is pungent and dispersing to promote the lung and bitter to lower the qi, which is the key medicine to promote the lung, open the coup, open the hairy orifices, promote the lung health, make the lung qi smooth, and restore the normal function of the lung division of suction and descent. Di Long is cold and descending, penetrating the upper and lower, good at enlightening the upper and declaring and lowering lung qi, draining lung heat and relieving cough and asthma, draining the lower, opening the state capital, and removing dampness and drenching [31]. The combination of the two drugs, one cold and one warm, one ascending and one descending, and the reasonable use of Xuan Dao and Tongluo, can make the evil of dampness and heat go away from the bottom. Bitter almonds, scape seeds, perilla seeds, and half-xia all have the effect of lowering qi, resolving phlegm, and relieving cough and asthma. Bitter almonds are bitter to lower the qi, moisten the stool, and warm to cathartic, while ephedra is pungent and dispersing, favoring the surface, and bitter almonds are bitter and descending, favoring the lining, which can restore the cathartic effect of lung qi and enhance the effect of ephedra in relieving cough and asthma. Daphne scabra is pungent and cold, smooth and downward, bitter and cold and subduing, and is specialized in dipping watery drinks and phlegm fire in the lung to calm cough and asthma. Perilla seeds are smooth and straight down and are mainly descending in nature, and are good at lowering lung qi and resolving phlegm and saliva; when qi is lowered and phlegm is eliminated, cough and asthma will be calmed. The combination of Radix Panax notoginseng, dampness, phlegm, and reversion can help Zizyphus to lower qi, resolve phlegm, and calm asthma, and the combination with almond can strengthen the function of suction. Scutellaria baicalensis, Morinda citrifolia, Qianhu, and Yujin are the adjuvants. Scutellaria baicalensis is bitter-cold in nature and enters the lung meridian to clear the heat in the upper jiao, so it is used with the pungent and warm Radix Panax notoginseng, which is used to clear heat and dispel phlegm [35]. The bitter cold of Scutellaria baicalensis and the warmth of Ephedra are mutually restrained, which enhances its effect on asthma without contributing to internal heat and does not cause the cold of Scutellaria baicalensis to deeply stagnate in the body and stagnate the qi, which can clear lung heat, dissolve phlegm and dampness, and relieve cough and asthma [36]. Mulberry bark, which is sweet in taste and cold in nature, can clear lung heat and relieve asthma as its main action. Mulberry bark, which can stabilize vital energy and compensate for deficiency by replenishing deficiencies, is usually used mainly to clear lung heat as well as relieve cough [37]. In combination with Scutellaria baicalensis, the heat-releasing power is even greater, and the sweet taste and cold nature of mulberry bark can counteract the bitter taste of Scutellaria baicalensis, clearing lung heat without harming Yin. Qian Hu descends Qi and dissolves phlegm, expels wind-heat, and is an important medicine for treating phlegm and Qi, and its use with ephedra's cold and heat can strengthen its power to expel lung heat [38]. It is pungent and can disperse, which can open the lung Jin's depression, release the depressed qi, and remove the fire evil then the cough will heal itself.

Our study is a retrospective randomized controlled study, and although it has some advantages in etiological inference, our study still has the following shortcomings. First, our study is a case-control study, not a randomized controlled trial, and is not blinded, so there is still some risk of bias; second, our study is a single-center clinical study, and the sample size included is small, and it still needs to be followed up by increasing the sample size and conducting multicenter. Finally, the clinical follow-up period of our study was relatively short, and long-term clinical follow-up is still needed.

In conclusion, the study of the clinical efficacy and low hospitalization cost of the self-prepared lung and asthma-restorative soup in patients with cough variant asthma significantly improved the patients' arterial oxygen saturation, acid-base value, arterial partial pressure of oxygen, and partial pressure of carbon dioxide and effectively controlled the heart rate and respiratory rate with high safety, which is worth further promotion.

## Figures and Tables

**Figure 1:** Evaluation of clinical efficacy; in our study, data on evaluation of clinical efficacy was statistically analyzed and calculated using SPSS 26.00 statistical software. The measured data were expressed as median, and the analysis of variance using repeated measures showed that patients underwent after Feidingchuan decoction; the heart rate, respiratory rate, blood arterial oxygen saturation, pH value, arterial blood oxygen partial pressure, and carbon dioxide partial pressure between the observation group and the reference group were significantly different between and within the group, with statistical differences (*P* < 0.05).

**Figure 2:** Treatment safety evaluation; in our study, data on treatment safety evaluation was statistically analyzed and calculated using SPSS 26.00 statistical software. The measured data were expressed as median, and the analysis of variance using repeated measures showed that with cough variant asthma, the drug toxicity and side effects of the patients after treatment showed that the red throat, shortness of breath, chest tightness, and dry mouth in the observation group were significantly different from those in the control group (*P* < 0.05).

**Figure 3:** Analysis of treatment benefit; in our study, data on treatment benefit analysis was statistically analyzed and calculated using SPSS 26.00 statistical software. The measured data were expressed as median, and the analysis of variance using repeated measures showed that after survey follow-up and statistics, the hospitalization time, hospitalization cost, asthma exacerbation control time, effective rate, and recurrence rate of the patients in the two groups were significantly different between and within the group (*P* < 0.05).

**Table 1:** Comparison of baseline data of two groups of patients.

Group	Average age (years)	Gender (men and women)	Common causes (*n* (%))				
			Exposure to allergens	Exposure to irritants	Allergic rhinitis	Respiratory infection	Premature withdrawal
Reference group (45)	47.91 ± 3.71	25/20	5 (11.11)	9 (20.00)	7 (15.56)	5 (11.11)	6 (13.33)
Observation group (45)	49.16 ± 5.62	22/23	8 (17.78)	6 (13.33)	4 (8.89)	6 (13.33)	9 (20.00)
*t*	-4.608	0.943	0.000				
*P*	0.115	0.445	1.000				

## Data Availability

No data were used to support this study.
